# Anticancer and Anti-Inflammatory Mechanisms of NOSH-Aspirin and Its Biological Effects

This article has been retracted.

**DOI:** 10.1155/2022/4463294

**Published:** 2022-08-17

**Authors:** Jun Zhou, Weihong Zeng, Ying Zeng, Yukun Li, Zheng Xiao, Juan Zou, Lijun Peng, Jiliang Xia, Xi Zeng

**Affiliations:** ^1^Hunan Province Key Laboratory of Tumor Cellular & Molecular Pathology, Cancer Research Institute, Hengyang Medical School, University of South China, Hengyang, Hunan 421001, China; ^2^School of Nursing, Hengyang Medical School, University of South China, Hengyang, Hunan 421001, China; ^3^Department of Spine Surgery, The First Affiliated Hospital, University of South China, Hengyang, Hunan 421001, China

## Abstract

NOSH-Aspirin, which is generated from NO, H_2_S, and aspirin, affects a variety of essential pathophysiological processes, including anti-inflammatory, analgesic, antipyretic, antiplatelet, and anticancer properties. Although many people acknowledge the biological significance of NOSH-Aspirin and its therapeutic effects, the mechanism of action of NOSH-Aspirin and its regulation of tissue levels remains obscure. This is in part due to its chemical and physical features, which make processing and analysis difficult. This review focuses on the biological effects of NOSH-Aspirin and provides a comprehensive analysis to elucidate the mechanism underlying its disease-protective benefits.

## 1. Introduction

The conventional treatment of cancer includes surgery, radiotherapy, chemotherapy, and biotherapy. Patients diagnosed with cancer at an early stage are most frequently treated surgically. While radiation therapy and chemotherapy have severe side effects on bone marrow hematopoietic cells, bone marrow hematopoietic cells are resistant to these treatments [1]. Targeted drugs are effective but have limited indications.

Aspirin, the most used nonsteroidal anti-inflammatory medication, exerts its antipyretic, analgesic, and anti-inflammatory actions by blocking prostaglandin synthesis [2]. As contemporary medicine has progressed, there is clinical evidence that aspirin can prevent colorectal, endometrial, ovarian, pancreatic, gallbladder, ureteral, gastric, and kidney cancers, as well as lower the incidence and spread of fibrosarcoma and prostate cancer [3–9]. However, long-term aspirin use can result in stomach ulcers, stomach bleeding, kidney failure, and other adverse effects [6, 10].

Hydrogen sulfide (H_2_S), one of three intracellular gaseous signal transducers, is essential to physiological activities [11]. It can influence the cell cycle, apoptosis, oxidative stress, neuronal and cardiovascular function, inflammation, and tumor formation [12–14]. According to several studies, greater concentrations of H_2_S (produced by an external H_2_S donor) inhibit tumor growth. In other studies [11, 15], we demonstrated that diallyl disulfide (DADS) suppresses gastric cancer *in vivo* and *in vitro*. However, the easy-volatile physical qualities of hydrogen sulfide make its application inconvenient.

Nitric oxide (NO), one of the three gaseous intracellular signal transducers, is an endogenously produced, short-lived signal molecule [16]. Currently, numerous NO donors have emerged as prospective therapeutic agents for cardiovascular and respiratory disorders, wound healing, immunological response to infection, and cancer [17]. However, its short half-life, chemical reactivity, fast systemic clearance, and cytotoxicity have impeded the clinical development of the vast majority of low-molecular-weight NO donors [18]. NO is dose and time dependent, just like H_2_S.

To overcome these restrictions, NO-NSAIDs and HS-NSAIDs were developed. Despite a considerable degree of stomach mucosal safety, the IC50 for growth inhibition of these two drugs [19, 20] is extremely high. And NO-NSAIDs produce quinone methide intermediates throughout the metabolic process, which calls into doubt the function of NO in their biological activity [20]. NOSH-Aspirin has eliminated the aforementioned two problems. This article will cover in detail the biological effects and mechanism of NOSH-Aspirin's protective effect against diseases and its biological effects.

## 2. The Physical and Physiological Characteristics of NOSH-Aspirin

NOSH-Aspirin has been available for roughly a decade. NOSH-Aspirin is derived from aspirin to which two groups releasing H_2_S and NO (Figure 1). According to the difference between the parent strains, it is further subdivided into four variations named NOSH-1, 2, 3, and 4. NOSH-1-3 are derived from salicylic acid, while NOSH-4 is derived from aspirin [21]. NOSH-1, on the other hand, processes three positional isomers: o-, m-, and p-NOSH-Aspirin [21, 22]. This article focuses mainly on o-NOSH-aspirin. NOSH-Aspirin is produced by combining aspirin, H_2_S, and NO. Therefore, it is reasonable to assume that NOSH-Aspirin shares three properties: It is slightly soluble in water, soluble in organic solvents, has a slight rotten egg odor, decomposes easily in the presence of light, and must be stored in the dark. Due to the long time it takes for NOSH-Aspirin to break down, H_2_S and NO are released gradually. In this way, the medicine can reach all of the cells and tissues in the body.

Studies have demonstrated that NOSH-Aspirin could be broken down into H_2_S, NO, and aspirin following ingestion. The amount of H_2_S and NO released is significantly more than that of NO-Aspirin and HS-Aspirin, extending the exposure of cells to H_2_S and NO [23]. And it also compensates for the high IC50 value of NO-Aspirin and HS-Aspirin in inhibiting growth [21, 24]. In addition, NOSH-Aspirin catabolism does not generate hazardous intermediates for the methylation of methyl benzoquinone [25]. In addition, the released H_2_S and NO enhance the mucosal defenses of the gastrointestinal tract [26–30]. NOSH-Aspirin enhances the safety of Aspirin and the impact of H_2_S and NO, regardless of the analysis.

## 3. The Biological Effects of NOSH-Aspirin

### 3.1. The Anti-Inflammatory Benefits of NOSH-Aspirin

Inflammation manifests itself clinically as redness, swelling, heat, discomfort, and dysfunction and is the body's defensive response to stimuli [31]. Cyclooxygenase (COX), also known as prostaglandin peroxidase synthase (PTGS), is the enzyme in charge of producing prostaglandins, prostacyclin, and thromboxane in the body [32]. COX is composed of two enzymes: intrinsic COX (COX-1) and inducible COX (COX-2). COX-1 interferes with the regulation of platelet aggregation, vascular movement, gastric mucosal blood flow, and renal blood flow [32], in order to maintain the stability of the physiological functioning of cells, tissues, and organs. Inflammation can encourage monocytes, macrophages, fibroblasts, etc. to produce COX-2, and the COX-2 production is a crucial step in triggering the subsequent inflammatory response. By decreasing COX, drugs can lessen the symptoms of inflammation and pain. Aspirin is among the most frequently used nonsteroidal anti-inflammatory drugs (NSAIDS) [33]. The majority of COX inhibitors are mostly nonsteroidal anti-inflammatory drugs. Aspirin exerts its antipyretic, analgesic, and anti-inflammatory effects by inhibiting the formation of prostaglandin (PG) synthesis [34].

According to studies, NOSH-Aspirin inhibits COX more effectively than aspirin. Due to inhibition of COX, the concentration of PGE2 is also decreased [35]. In addition, it suppresses the writhing response and hypercoagulation produced by inflammation in a dose-dependent manner, lowers the generation and release of IL-1*β* during the inflammatory phase, and could lessen the nerve inflammation caused by the activation of microglia and astrocytes [36]. Moreover, it also has superior protective effects to NO-Aspirin and HS-Aspirin [24, 35, 37, 38]. Consequently, it is also considered as a potential novel treatment for neurodegenerative diseases [39]. According to analysis, aspirin can reduce brain inflammation; H_2_S can eliminate heavy metals from plaques; and NO can widen blood vessels, reduce inflammation, and boost oxygen delivery to neurons. In addition, NOSH-Aspirin increases anti-inflammatory drugs, making it more effective.

### 3.2. NOSH-Aspirin Has anti-Cancer Properties

#### 3.2.1. NOSH-Aspirin Inhibits COX to Fight Tumors

Numerous cancer cell growth and apoptosis have been linked to COX targets [40]. Currently, inhibitors of mature COX targets such as Celocoxib [41], Diciofenac [32], and Ginsenoside [42] are being investigated. COX-2 is usually overexpressed in epithelial malignancies, including breast, prostate, lung, kidney, ovarian, and liver cancers, and this overexpression can lead to deterioration [43–48]. COX-2 inhibition could help prevent of colon, lung, breast, pancreatic, and skin cancer. A variety of cancer cells express COX2, which is associated with a poor prognosis. It has been shown that the main enzyme of PEG2 can increase tumor cell growth, proliferation, and metastasis and that PEG2 in the tumor microenvironment actively promotes tumor immune evasion in a variety of ways, resulting in suboptimal immunotherapy outcomes.

Researchers have found that NOSH-Aspirin can decrease the expression of COX1 and COX2 [22, 24, 49]. We hypothesize that NOSH-Aspirin inhibits COX mainly through its breakdown product, aspirin. Epidemiological studies indicate that NSAIDs are frequently used as chemopreventive agents for several forms of cancer. Studies have indicated that NASIDs reduce colon cancer incidence and mortality by 50% [50]. NOSH-Aspirin inhibits COX in the liver, colon, pancreas, lung, prostate, breast, and leukemia without the toxicity and side effects associated with NSAIDs [21, 24, 36–38, 49]. COX-1 and COX-2 deficiency has been shown in studies to reduce the number and formation of intestinal tumors in mice. In vivo, NOSH-Aspirin inhibits COX more effectively than aspirin alone, and it is dose- and time-dependent [21]. This series of studies suggests that NOSH-Aspirin inhibits cancer by blocking COX.

#### 3.2.2. Tumor Growth Inhibition by NOSH-Aspirin

Tumors are diseases characterized by uncontrolled cell growth and multiplication as a result of abnormal cell growth, differentiation and death. Among these, disruption of the cell cycle is the most important cancer process [51]. The discovery of maturation-stimulating factors, cell cycle proteins, and cell cycle-dependent protein kinases further confirmed a close association between the cell cycle and cancer development.

NOSH-Aspirin inhibits G0/G1 cell cycle arrest in both colon cancer and pancreatic cancer cell lines [24, 49, 52]. Furthermore, it was discovered that NOSH-Aspirin can simultaneously inhibit FOXM1 [49]. FOXM1 is a Forkhead family tumorigenic transcription factor that has been found to play an important role in the proliferation and cell cycle development of numerous tumor cell types [53]. FOXM1 is associated with cell proliferation. It increases cell proliferation primarily by inhibiting cell cycle-dependent kinase inhibitors, but it also plays a function in growth hormone-mediated cell proliferation [53]. FOXM1 overexpression in numerous malignant tumor cell lines may be a necessary proto-oncogene for tumor growth.

In addition, cells treated with NOSH-Aspirin showed reduced expression of PCNA [23]. PCNA is a co-factor of DNA polymerase delta and can respond to DNA damage during DNA replication. PCNA is only seen in proliferating cells and tumor cells [54]. It is further suggested that NOSH-Aspirin reduces the growth of tumor cells by inhibiting FOXM1 and PCNA.

#### 3.2.3. NOSH-Aspirin Induces Tumor Apoptosis

Apoptosis is a type of programmed cell death, which is actively implemented by cells and is generally caused by physiological or pathological circumstances. Typically, cancer cells usually have anti-apoptosis mechanisms. The use of apoptosis mechanisms to treat tumors is to change the balance between pro-apoptosis and anti-apoptosis at all levels of apoptosis regulation, induce tumor cell apoptosis, and achieve anti-apoptosis [51]. NOSH-Aspirin promotes anti-cancer effects by targeting tumor necrosis factor a (TNF-*α*), Fas-FasL system, tumor necrosis factor-related apoptosis-inducing ligand TRAIL, and targeting Bcl-2 protein family, NF-*κ*B, and caspase, etc. [55].

Prior research has demonstrated that NOSH-Aspirin can induce tumor apoptosis [38, 56]. Additional research has shown that it can increase the intracellular TNF-*α*, increase the activity of caspase-3, and inhibit the expression of NF-*κ*B [49, 57, 58]. Experiments in vivo and in vitro have shown that TNF-*α* has a powerful effect of inducing apoptosis and caspase-3 can increase the induction of death receptors or the induction of radiotherapy and chemotherapy to increase the sensitivity of apoptosis [49]. There are many anti-apoptotic proteins in the downstream genes of NF-*κ*B, such as Bcl-2, Bcl-XL, Bfl-1, cIAP1, cIAP2, TRAF1, and TRAF2. NF-*κ*B inhibits these anti-apoptotic proteins by inducing or upregulating Apoptosis, and it has also been reported that NF-*κ*B can promote the expression of Fas, FasL, DR4, and DR5 and promote apoptosis in some specific cases, but in general, the constitutive activation of NF-*κ*B helps tumor cells to escape apoptosis [59]. The pro-apoptotic activity of NOSH-Aspirin is undoubtedly a new route for the research of antitumor drugs. Literature has shown that while promoting apoptosis, it will also increase the sensitivity of tumor cells to radiotherapy and chemotherapy [60]. This also suggests a new direction for whether NOSH-Aspirin could be used as a radiation and chemotherapy adjuvant. Therefore, we believe that NOSH-Aspirin could inhibit NF-*κ*B and promote TNF-*α* and Caspase-3 to exert anti-tumor actions.

#### 3.2.4. NOSH-Aspirin Increases Intracellular ROS

Reactive oxygen species (ROS) is a collection of short-lived, highly reactive oxygen-containing molecules that can cause DNA damage and influence the DNA damage response (DDR) [61]. In general, tumor cells employ diverse defense mechanisms to mitigate the deleterious effects of ROS, thereby maintaining a relative equilibrium in the generation and removal of ROS, which is crucial for their survival. It is currently assumed that ROS plays a dual role in malignancies. On the one hand, ROS can activate a variety of redox reactions and signaling pathways, such as the MAPK pathway, PI3K/AKT pathway, NF-*κ*B pathway, and Keap1-Nrf2-ARE pathway, to promote tumor occurrence, development, and metastasis; on the other hand, when ROS exists in excess, it can cause cellular stress and damage through oxidative stress mechanism and eventually lead to cell death [62–64]. It all depends on the severity of the ROS excess and the duration of exposure; oxidative stress can activate cell survival or apoptosis mechanisms. At low concentrations, ROS may function as signal transduction molecules that promote tumorigenesis and heterogeneity, while at high concentrations, cancer cells may be harmed, become genotoxic, or undergo apoptosis.

Vannini and Chattopadhyay discovered that NOSH-Aspirin could generate ROS levels in cancer cells in a dose-dependent manner [22, 56]. Despite being minimally differentiated, cancer cells lack the ability to fight free radicals. When the generation of reactive oxygen species (ROS) and the endogenous antioxidant defense mechanism are out of balance, oxidative stress will occur in the cell, which will eventually lead to cell death. In addition, in pancreatic cancer cells lacking P53, their cell growth is strongly inhibited by ROS-inducing compounds [49]. In addition, it has been reported that pancreatic cancer cells with lower ROS levels are more resistant to chemotherapy. This may be attributed to the synergistic effect of HS-Aspirin and NO-Aspirin.

#### 3.2.5. Other Biological Effects

In addition to its anti-inflammatory and anticancer activities, NOSH-Aspirin also exhibits antipyretic, analgesic, antiplatelet, and reducing oxidative stress-reducing biological actions [56]. These biological effects are tissues and organism-protective.

## 4. Perspectives

Cancer is the leading cause of death in every country on earth and a significant barrier to extending life expectancy. According to World Health Organization (WHO) estimates in 2018, cancer is the second or second largest cause of mortality [65]. According to Global Cancer Statistics 2020, female breast cancer has surpassed lung cancer as the most common cancer, followed by lung cancer (11.4%), colorectal cancer (10.0%), and prostate cancer (7.3%) [66]. Moreover, pancreatic cancer and leukemia were rated fourteenth and fifteenth, respectively. Therefore, it is of the utmost importance to investigate novel anticancer medications.

NOSH-Aspirin is a super aspirin that can provide H_2_S, NO, and aspirin at the same time, with the potential to suppress colon, breast, pancreatic, lung, and prostate cancer, as well as leukemia. Compared to aspirin, this chemical protects the stomach mucosa and enhances the anticancer and anti-inflammatory activities of aspirin, H2S, and NO. NOSH-Aspirin is exceedingly safe and has no effect on normal epithelial cells. By regulating intracellular ROS, suppressing inflammation, inhibiting COX, inhibiting NF-B, activating caspase-3, and decreasing FoxM1 expression, NOSH-Aspirin can cause cell apoptosis, decrease proliferation, and stop the cell cycle [21, 24, 36–38, 49, 58]. Furthermore, it was discovered that NOSH-Aspirin reduced the expression of *β*-catenin in cells, suggesting that it may also affect the WNT signaling pathway. NOSH-Aspirin can raise blood pressure. NOSH-Aspirin can raise cellular iNOS levels [49] (Figure 2). The presence of iNOS in the cell enhances the cytotoxic action of NO, resulting in a more potent antitumor effect. NOSH-Aspirin is effective against six types of cancer, including colon cancer, breast cancer, pancreatic cancer, lung cancer, bladder cancer, and leukemia. The tumor volume of mice treated with NOSH-Aspirin was significantly reduced in the xenograft model when compared to untreated mice [24, 49]. In addition to suppressing tumors, it has been discovered that the anti-inflammatory effect of NOSH-Aspirin has a protective effect in Alzheimer's disease [39].

Despite the aforementioned advantages, NOSH-Aspirin has a number of disadvantages. More research is needed to confirm the NOSH-Aspirin target and specific signaling pathways. Although NOSH-Aspirin does not destroy normal epithelial cells, little is known about its toxicity and side effects on the hematological system, liver, and other organs. Because it is unknown whether NOSH-Aspirin can be combined with other chemotherapy or targeted medications. We are unaware of whether NOSH-Aspirin is used alone or in combination with other drugs to treat tumors. Large-scale clinical trials to confirm its feasibility in cancer treatment are still lacking.

## 5. Conclusions

Overall, the development and implementation of NOSH-Aspirin-based cancer treatment methods is still in its infancy. Future practical application of NOSH-Aspirin as a more effective cancer treatment will require additional investigation.

## Figures and Tables

**Figure 1:** The spatial structure of NOSH compounds. The gray is the parent compound—aspirin. ADT-OH (5-(4-hydroxyphenyl)-3H-1,2-dithio-3-thione) which releases H_2_S is in the blue. The pink is the nitrate group that releases NO.

**Figure 2:** NOSH-Aspirin regulates the several molecular thus to protect mucosa membrane and inhibit multiple cancer.

## Data Availability

The data used to support the findings of this study are available from the corresponding author upon request.
